# Value of CSF-Cl, CSF-GS, CSF-MALB, and CSF-ADA in Differential Diagnosis of Secondary Hydrocephalus

This article has been retracted.

**DOI:** 10.1155/2022/6742795

**Published:** 2022-05-28

**Authors:** Junzhang Huang, Bing Chen

**Affiliations:** Department of Neurosurgery, Guangdong Medical University, Zhanjiang City, Guangdong Province, China

## Abstract

**Objectives:**

To investigate the value of cerebrospinal fluid chloride (CSF-Cl), cerebrospinal fluid glucose (CSF-GS), cerebrospinal fluid microalbumin (CSF-MALB), and cerebrospinal fluid adenosine deaminase (CSF-ADA) in the differential diagnosis of secondary hydrocephalus.

**Methods:**

103 patients with secondary hydrocephalus treated in our hospital from January 2018 to April 2022 were selected. According to different types, it is divided into the hemorrhagic hydrocephalus group and tumor hydrocephalus group. By detecting the levels of inflammatory factors such as CSF-Cl, CSF-GS, CSF-MALB, and CSF-ADA in the two groups, we can analyze the value of these inflammatory factors in the differential diagnosis of secondary hydrocephalus.

**Results:**

The level of CSF-MALB in the hemorrhagic hydrocephalus group was significantly higher than that in the tumor hydrocephalus group, and the difference between the two groups was statistically significant (*P* < 0.05). There was no significant difference in the levels of CSF-Cl, CSF-GS, and CSF-ADA between the two groups (*P* > 0.05). The area under ROC curve (AUC) of CSF-Cl, CSF-GS, CSF-MALB, and CSF-ADA in the differential diagnosis of secondary hydrocephalus was 0.438, 0.553, 0.750, and 0.542, respectively, sensitivity was 15.1%, 45.3%, 79.2%, and 18.9%, respectively, and specificity was 96.0%, 80.0%, 80.0%, and 94.0%, respectively.

**Conclusions:**

The inflammatory reaction of hemorrhagic hydrocephalus was significantly greater than that of tumor hydrocephalus. Moreover, CSF-MALB is closely related to the pathogenesis of hemorrhagic hydrocephalus. At the same time, CSF-MALB can be used as a good index for rapid differential diagnosis of secondary hydrocephalus.

## 1. Introduction

Secondary hydrocephalus is a common critical disease in neurosurgery. It often has the characteristics of acute onset, rapid progress, many complications, and high disability rate [1]. If the treatment is not timely, it may lead to lifelong disability, leaving irreversible damage, and even endanger the life and health of patients [2, 3]. Hemorrhagic hydrocephalus and neoplastic hydrocephalus are two common types of secondary hydrocephalus [3, 4]. Early diagnosis of secondary hydrocephalus is of great significance to guide clinical treatment and improve the prognosis of patients [5, 6]. We used to rely on typical symptoms and signs and imaging examination to distinguish between hemorrhagic hydrocephalus and neoplastic hydrocephalus [7, 8]. However, some patients may have no specific symptoms and signs, and the imaging changes are often not obvious, which leads to the difficulty of clinical diagnosis and treatment [9, 10].

Some studies have shown that there are differences in the expression of some inflammatory indexes in different neurosurgical diseases [11, 12]. Detecting these inflammatory indicators can help us quickly identify the types of secondary hydrocephalus, so as to guide our clinicians to take reasonable and effective treatment measures to better improve the quality of life and prognosis of patients [13, 14]. Cerebrospinal fluid chloride (CSF-Cl), cerebrospinal fluid glucose (CSF-GS), cerebrospinal fluid microalbumin (CSF-MALB), and cerebrospinal fluid adenosine deaminase (CSF-ADA) are recently considered to be inflammatory markers associated with nervous system injury.

Laboratory tests are the gold standard for surgical diagnosis. We expect to identify different types of hydrocephalus through these laboratory inflammatory factors. However, there are few studies on this aspect at present. At present, there are few studies on the inflammatory indexes of cerebrospinal fluid chloride (CSF-Cl), cerebrospinal fluid glucose (CSF-GS), cerebrospinal fluid microalbumin (CSF-MALB), and cerebrospinal fluid adenosine deaminase (CSF-ADA) in the literature at home and abroad [15, 16]. The mechanism of these indexes in secondary hydrocephalus is not very clear [17, 18]. This study compared the levels of CSF-Cl, CSF-GS, CSF-MALB, and CSF-ADA between the hemorrhagic hydrocephalus group (H-HCP group) and tumor hydrocephalus group (T-HCP group) from January 2018 to April 2022 to explore the value of these four indicators in the differential diagnosis of secondary hydrocephalus, so as to provide clinical data support for the diagnosis and treatment of secondary hydrocephalus [19, 20]. The inflammatory reaction of hemorrhagic hydrocephalus was significantly greater than that of tumor hydrocephalus. Moreover, CSF-MALB is closely related to the pathogenesis of hemorrhagic hydrocephalus. At the same time, CSF-MALB can be used as a good index for rapid differential diagnosis of secondary hydrocephalus.

## 2. Materials and Methods

### 2.1. Study Design

103 patients with secondary hydrocephalus treated in the Affiliated Hospital of Guangdong Medical University from January 2018 to April 2022 were selected. According to different etiological types, they were divided into the hemorrhagic hydrocephalus group (H-HCP group, *n* = 53) and tumor hydrocephalus group (T-HCP group, *n* = 50). There were 25 males and 28 females in the H-HCP group, aged 12–83 years, with an average age of 54.1 years. There were 17 males and 33 females in the T-HCP group, aged 2–73 years, with an average age of 36.9 years. There was no significant difference in gender, age, and course of disease between the two groups. Inclusion criteria were as follows: it meets the diagnostic criteria of hemorrhagic hydrocephalus and tumor hydrocephalus; CT or MRI showed enlargement of the ventricular system; the patients had no diseases such as cardiopulmonary disease and diabetes; and the patient's clinical data are complete. Exclusion criteria were as follows: the patient has heart lung disease or diabetes; the patient does not cooperate with the treatment or cannot perform lumbar puncture; and the patient's clinical data are incomplete.

### 2.2. Methods

The patient underwent lumbar puncture on the second day after admission. Determine the puncture point and take the intersection of the connecting line of the highest point of bilateral iliac crest and the posterior midline at the puncture point. We assist the patient to set the body position. Generally, the patient has an obligation to take the lateral position, bend the hip and knees, excessively bend the neck, hold the knees with both the hands, and completely expose the waist. The place should be disinfected and sealed with towels. The puncture point should be anesthetized layer by layer. Use the puncture needle to slowly enter the needle until the needle feels empty and then pull out the needle core and see cerebrospinal fluid dripping out. At this time, quickly measure the pressure of cerebrospinal fluid and reserve 6 ml of cerebrospinal fluid sample for the relevant examination. Then, slowly pull back the needle, cover the puncture site with gauze, and fix it with adhesive tape. The patient is obliged to go to the pillow and lie flat for more than six hours. Transfer 6 ml of cerebrospinal fluid sample to 1.5 ml of a sterile EP tube, centrifuge, discard cells and tissue precipitation, collect supernatant, and store the collected supernatant in a refrigerator at −80°C for examination. We used MALB reagent and latex immunoturbidimetry to determine the level of CSF-MALB.

### 2.3. Statistical Analysis

The study used SPSS statistical software for data analysis. The counting data were analyzed by the chi-square test and Fisher exact probability method. The measurement data are expressed as mean ± standard deviation, and the measurement data of two independent samples are tested by the *t*-test. By drawing the receiver operating curve (ROC), we analyzed the value of CSF-Cl, CSF-GS, CSF-MALB, and CSF-ADA in the differential diagnosis of secondary hydrocephalus. *P* < 0.05 was statistically significant.

## 3. Results

### 3.1. Comparison of CSF-Cl, CSF-GS, CSF-MALB, and CSF-ADA between the Two Groups

In the H-HCP group, the expression level of CSF-MALB was 530.24 ± 319.23 mg/L. In the T-HCP group, the expression level of CSF-MALB was 318.82 ± 353.81 mg/L. CSF-MALB in the H-HCP group was significantly higher than that in the T-HCP group, and the difference between the two groups was statistically significant (*P* < 0.05). There was no significant difference in CSF-Cl, CSF-GS, and CSF-ADA between the two groups (*P* > 0.05) (Table 1).

### 3.2. Value of CSF-Cl, CSF-GS, CSF-MALB, and CSF-ADA in Differential Diagnosis of Secondary Hydrocephalus

The area under ROC curve (AUC) of CSF-Cl, CSF-GS, CSF-MALB, and CSF-ADA in the differential diagnosis of secondary hydrocephalus was 0.438, 0.553, 0.750, and 0.542, respectively, sensitivity was 15.1%, 45.3%, 79.2%, and 18.9%, respectively, and specificity was 96.0%, 80.0%, 80.0%, and 94.0%, respectively (Table 2, Figure 1).

## 4. Discussion

The treatment plan and prognosis of secondary hydrocephalus are related to different causes [21, 22]. Early identification of the types of secondary hydrocephalus is of great significance to control the stability of the disease and improve the prognosis [23, 24]. The clinical diagnosis of hemorrhagic hydrocephalus and neoplastic hydrocephalus sometimes does not completely depend on the symptoms, signs, and imaging manifestations, but the detection of cerebrospinal fluid can not only improve the diagnostic accuracy of secondary hydrocephalus but also quickly help our clinical workers quickly evaluate the severity of the patient's condition [25, 26].

The normal value of CSF-Cl is the normal value of the chloride content in cerebrospinal fluid and the reference range of the normal value of chloride in cerebrospinal fluid [27, 28]. Calculated by NaCl, 110–122 mmol/L for infants; children 117–127 mmol/L; adult 119–129 mmol/L. Under normal conditions, all substances between blood and cerebrospinal fluid cannot enter and leave the circulation freely. When some diseases involve the central nervous system, the chloride content in cerebrospinal fluid will change. As a specific indicator of secondary hydrocephalus inflammation, its mechanism is not very clear. By comparing the H-HCP group and T-HCP group, we found that there was no significant difference between them (*P* > 0.05). At the same time, we found that AUC was 0.438 (ACU <0.7), sensitivity was only 15.1%, and specificity was 96.0%. This shows that the accuracy of CSF-Cl in the diagnosis of secondary hydrocephalus is not high, and its sensitivity is not strong, which is inconsistent with the standard that we need to screen different types of secondary hydrocephalus. CSF-Cl cannot quickly distinguish hemorrhagic hydrocephalus from neoplastic hydrocephalus.

The normal value of CSF-GS is 2.5–4.4 mmol/L [29, 30]. The content of sugar in cerebrospinal fluid depends on the level of blood glucose. The normal value is usually 50%–70% of blood glucose. Cerebrospinal fluid examination is an important means for clinical diagnosis of central nervous system infection, cerebrospinal fluid leakage, hydrocephalus, increased cerebrospinal fluid pressure, and meningeal carcinomatosis. The role of CSF-GS in the occurrence of secondary hydrocephalus is unclear, but its value often increases. By comparing the H-HCP group and T-HCP group, we found that there was no significant difference between them. The AUC of CSF-GS was 0.553 (AUC <0.7), sensitivity was only 45.3%, and specificity was 80.0%. This side reflects the low accuracy and sensitivity of CSF-GS in identifying the types of secondary hydrocephalus. CSF-GS cannot distinguish hemorrhagic hydrocephalus from neoplastic hydrocephalus.

CSF-MALB is a sensitive index and specific inflammatory factor in the early stage of blood-brain barrier permeability change and participates in the process of immune regulation. When the blood-brain barrier is destroyed, cerebrospinal fluid microalbumin is very easy to enter cerebrospinal fluid from blood by relying on a large concentration difference. Therefore, it has high sensitivity and can be used as a specific evaluation index for the initial change of blood-brain barrier permeability. The results of this study showed that there were differences in CSF-MALB levels between the hemorrhagic hydrocephalus group and tumor hydrocephalus group. The level of CSF-MALB in the hemorrhagic hydrocephalus group was significantly higher than that in the tumor hydrocephalus group. The difference between the two groups was statistically significant. It shows that hemorrhagic hydrocephalus destroys the blood-brain barrier more than tumor hydrocephalus, and the inflammatory response of hemorrhagic hydrocephalus is greater than tumor hydrocephalus. Therefore, the level of CSF-MALB in cerebrospinal fluid will be greater. The AUC was 0.750 (AUC >0.7), sensitivity was 79.2%, and specificity was 80.0%. It shows that CSF-MALB has certain accuracy in diagnosing the types of secondary hydrocephalus, and its sensitivity and specificity are high. It can be used as a biochemical measurement index to distinguish the two types of secondary hydrocephalus: bloody hydrocephalus and tumor hydrocephalus.

CSF-ADA is an important enzyme in the purine nucleoside metabolism. CSF-ADA is a sensitive index reflecting brain injury. It can be used as one of the routine examination items of brain function and can reflect the enzymatic changes of central nervous system function. In the process of secondary hydrocephalus, CSF-ADA is also one of the specific indicators of inflammation in secondary hydrocephalus. By comparing the HCP group and CSF-ADA group, we found that there was no significant difference between them. The AUC of CSF-ADA was 0.542 (AUC <0.7), sensitivity was 18.9%, and specificity was 94.0%. This shows that CSF-ADA is not accurate in distinguishing the types of secondary hydrocephalus, and its sensitivity is not high. It cannot be used as a biochemical measurement index to distinguish hemorrhagic hydrocephalus and neoplastic hydrocephalus.

In conclusion, the inflammatory reaction of hemorrhagic hydrocephalus was significantly greater than that of tumor hydrocephalus. CSF-MALB is involved in the change of disease mechanism of secondary hydrocephalus. The detection of the CSF-MALB level can provide a basis for the early identification of the types of secondary hydrocephalus and the evaluation of the disease, which is helpful to guide the clinical medication and surgical treatment.

## Figures and Tables

**Figure 1:** ROC curve of differential diagnosis of CSF-Cl, CSF-GS, CSF-MALB, and CSF-ADA.

**Table 1:** Comparison of CSF-Cl, CSF-GS, CSF-MALB, and CSF-ADA (*n* = 53 in the H-HCP group; *n* = 50 in the T-HCP group).

Groups	CSF-Cl (mmol/L)	CSF-GS (mmol/L)	CSF-MALB (mg/L)	CSF-ADA (U/L)
H-HCP group	115.15 ± 17.50	3.46 ± 1.27	530.24 ± 319.23	2.33 ± 4.52
T-HCP group	117.63 ± 18.23	3.18 ± 1.04	318.82 ± 353.81	1.92 ± 2.65
*T* value	−0.704	1.223	3.187	0.557
*P* value	0.483	0.224	0.002^*∗*^	0.574

H-HCP group, hemorrhagic hydrocephalus group; T-HCP group, tumor hydrocephalus group. ^*∗*^*P* < 0.05.

**Table 2:** Value of CSF-Cl, CSF-GS, CSF-MALB, and CSF-ADA in differential diagnosis of secondary hydrocephalus.

Item	Cutoff value	Sensitivity %	Specificity %	Youden index	AUC	95% CI
CSF-Cl	128.60 mmol/L	15.1	96.0	0.111	0.438	0.325–0.550
CSF-GS	3.75 mmol/L	45.3	80.0	0.253	0.553	0.439–0.667
CSF-MALB	300.30 mg/L	79.2	80.0	0.592	0.750	0.649–0.851
CSF-ADA	3.35 U/L	18.9	94.0	0.129	0.542	0.430–0.653

## Data Availability

The data used to support the findings of this study are available from the corresponding author upon request.
